# Central extracorporeal life support with left ventricular decompression for the treatment of refractory cardiogenic shock and lung failure

**DOI:** 10.1186/1749-8090-9-60

**Published:** 2014-03-29

**Authors:** Alexander Weymann, Bastian Schmack, Anton Sabashnikov, Christopher T Bowles, Philipp Raake, Rawa Arif, Markus Verch, Ursula Tochtermann, Jens Roggenbach, Aron Frederik Popov, Andre Ruediger Simon, Matthias Karck, Arjang Ruhparwar

**Affiliations:** 1 Department of Cardiothoracic Transplantation & Mechanical Circulatory Support, Royal Brompton and Harefield NHS Foundation Trust, Hill End Road, Harefield, Middlesex, UB9 6JH London, UK; 2 Department of Cardiac Surgery, Heart Center - University of Heidelberg, INF 110, 69120 Heidelberg, Germany; 3 Department of Cardiology, Angiology and Pulmonology, Heart Center – University of Heidelberg, INF 410, 69120 Heidelberg, Germany; 4 Department of Anesthesiology, University of Heidelberg, INF 110, 69120 Heidelberg, Germany; 5 Department of Thoracic and Cardiovascular Surgery, University Hospital Göttingen, Robert-Koch-Straße 40, 37075 Göttingen, Germany

**Keywords:** Mechanical circulatory support, Cardiogenic shock, Lung failure, Extracorporeal life support

## Abstract

**Background:**

The purpose of this prospective study was to evaluate the effects and functional outcome of central extracorporeal life support (ECLS) with left ventricular decompression for the treatment of refractory cardiogenic shock and lung failure.

**Methods:**

Between August 2010 and August 2013, 12 consecutive patients (2 female) with a mean age of 31.6 ± 15.1 years received central ECLS with left ventricular decompression for the treatment of refractory cardiogenic shock and lung failure. Underlying disease was acute cardiac decompensation due to dilated cardiomyopathy (n = 3, 25%), coronary artery disease with acute myocardial infarction (AMI) (n = 3, 25%), and acute myocarditis (n = 6, 50%). We routinely implemented ECLS by cannulating the ascending aorta, right atrium and inserting a left ventricular decompression cannula vent via the right superior pulmonary vein.

**Results:**

All patients were successfully bridged to either recovery (n = 3, 25%), long-term biventricular support (n = 6, 50%) or cardiac transplantation (n = 3, 25%). Seven patients (58.3%) were discharged after a mean hospital stay of 42 ± 11.9 days. The overall survival from ECLS implantation to the end of the study was 58.3%. The cumulative ICU stay was 23.1 ± 9.6 days. The length of support was 8.0 ± 4.3 days (range 3-17 days).

**Conclusions:**

We strongly recommend left ventricular decompression in refractory cardiogenic shock and lung failure to avoid pulmonary edema, left heart distension and facilitate myocardial recovery.

## Background

Cardiogenic shock still has an unfavorable prognosis with a mortality rate of 50-80% [1-4]. The prognosis strongly depends on the delay between the compromise and reestablishment of adequate end-organ perfusion. Analysis of the Interagency Registry for Mechanically Assisted Circulatory Support (INTERMACS) reveals that the proportion of INTERMACS level 1 patients (cardiogenic shock) undergoing long term VAD therapy has decreased from 42% in 2006 to 14% in 2012 due to poor outcomes. This has provided impetus to implement a more effective support strategy, which increasingly is taking the form of a bridge to bridge (salvage) approach using temporary extracorporeal devices in the first instance. Once the patient has been stabilised and has recovered end-organ function, replacement with a long-term support device can be considered [5].

Extracorporeal Life Support (ECLS) is an indispensable therapy for the acute treatment of patients with cardiogenic shock with or without lung failure. A common problem observed during ECLS is the absence of left heart decompression, which frequently leads to pulmonary edema and left ventricular distension which if untreated can cause subendocardial ischemia.

The purpose of our study was to objectively evaluate our institutional experience of left heart unloading during ECLS using a left ventricular vent with the aim of developing appropriate clinical management strategies and improving outcomes in this patient group.

## Methods

### Study design and patient cohort

A single arm, prospective study design was approved by our Institutional Review Board (Medical faculty of the University of Heidelberg). Patient demographics, preoperative medical history, operative and post-operative course data were collected from hospital medical records. Baseline demographics are presented in Table 1. Between August 2010 and August 2013 in our institution, 12 consecutive (2 female) patients (aged 31.6 ± 15.1 years, range 12-65 years) underwent ECLS with left ventricular decompression as a salvage procedure. The underlying pathological condition was refractory cardiogenic shock and lung failure in all study subjects (Figures 1 and 2). Cardiogenic shock was defined as a cardiac index (CI) lower than 2.2 liters/min/m^2^, systolic pressure lower than 90 mmHg for more than 30 minutes and clinical signs of hypoperfusion (cold extremities, oliguria or altered mental state) refractory to fluid resuscitation and intravenous inotropic support. Respiratory failure was defined as acute hypoxemia refractory to protective lung strategy ventilation for acute lung injury or equivalent (P_a_O_2_ < 8.0 kPa, P_a_CO_2_ > 6.7 kPa, pH < 7.2 at FiO_2_ 1.00).

**Table 1:** Baseline characteristics

**Baseline variables**	**n = 12**
Age, years	31.6 ± 15.1
Female sex	2 (16,7%)
CardioHelp system	2 (16.7%)
Cardiovascular risk factors	
Coronary heart disease	3 (25%)
Pulmonary Hypertension > 60 mmHg sys.	3 (25%)
LVEF before MCS, %	12.5 ± 5.4
Intra-aortic balloon pump	3 (25%)
Mechanical ventilation	12 (100%)
Pneumonia	2 (16.7%)
Pankreatitis	1 (8.3%)
Sepsis	3 (25%)
Renal failure	8 (66.7%)
Liver failure	10 (83.3%)
Cardiac arrest > 30 min	6 (50%)
HIT	2 (16.7%)

*LVEF*, Left ventricular ejection fraction; *HIT*, Heparin-induced thrombocytopenia.

**Figure 1:** **Clinical images from a representative patient of our study cohort: Left – Endotracheal tube with overflowing secretions, Right – Transesophageal echocardiography demonstrating dilated left ventricle with stasis despite peripheral ECMO support (CardioHelp™-System, Maquet, Rastatt, Germany) on admission.**

**Figure 2:** **Anteroposterior chest x-ray of a typical patient of our study cohort with cardiogenic shock before (A) and after (B) initiation of ECLS with left ventricular decompression.** The system rapidly induces a significant decrease in pleural effusion and pulmonary congestion.

### Surgical technique

A median sternotomy surgical approach was selected for all patients in the expectation of potential upgrade to long-term mechanical circulatory support. A 22 Fr. arterial cannula (Edwards Lifesciences Corporation, Irvine, USA) was inserted using the Seldinger technique into the distal ascending aorta, and the right atrium was cannulated for venous return with a 28 Fr. cannula of adjustable conformation (Medtronic, Minneapolis, USA) which was oriented prior to insertion such that its tip was directed towards the tricuspid valve. A heparin-coated 24 Fr. venting cannula (Medtronic, Minneapolis, USA), similarly pre-oriented, was inserted through the right superior pulmonary vein into the left ventricle and was connected to the ECLS inflow (venous drainage) using a Y-connector (Figure 3). The ECLS system consisted of a Levitronix CentriMag blood pump (Levitronix LLC, Waltham, Massachusetts, United States of America), a D902 ECMO oxygenator (Dideco, Sorin Group, Milan, Italy) and phosphorylcholine P.h.i.s.i.o-coated circuit tubing (Sorin Group, Milan, Italy). The maximum flow rate through the vent cannula depends primarily on its diameter and to a lesser extent its length.

**Figure 3:** **3-D reconstruction of left ventricular decompression using a vent implanted via the right superior pulmonary vein (A) through the mitral valve (B) into the left ventricle.** RA: right atrium; SVC: superior vena cava; PV: right superior pulmonary vein, LV: left ventricular.

The targeted extracorporeal support flow was 2.6 L/min/m^2^ body surface area for all patients. Intra-operative transesophageal echocardiography (TEE) was routinely performed to confirm correct positioning of the cannulas and this technique was repeatedly applied postoperatively to confirm adequate left ventricular decompression. ECLS total blood flow and left heart vent blood flow were monitored continuously using ultrasonic probes (Transonics Inc.) and continous brain oximetry (near-infrared spectroscopy, INVOS™) was monitored during the Intensive Care Unit (ICU) stay. A three-way tap was routinely placed in the proximal venous line and in the left ventricular vent line (Figure 4). This allowed separate blood gas analyses to be performed in each line and assisted in the detection of coronary hypoxia if the left ventricle began to recover.

**Figure 4:** **Setup of the presented circuit on intensive care unit.** RA indicates right atrium, LV left ventricle and Ao ascending aorta. The arrows indicate the direction of blood flow. The three-way taps are used for blood sampling to measure pre-pulmonary mixed venous oxygen saturation and post-pulmonary arterial oxygen saturation. Thus, the effectiveness of the circuit can be monitored continuously and accurately.

The ECLS weaning procedure consisted of intermittently reducing the blood flow rate, having ascertained that the left ventricle was not akinetic. This not only increased the left ventricular preload but also decreased its afterload, thereby facilitating left ventricle ejection. The feasibility of weaning from ECLS was evaluated by clinical judgment and transesophageal echocardiography at a reduced pump flow after a minimum of 48 hours’ support. All patients underwent daily TEE investigations, and procedural success was defined as a sustained reduction in left ventricular dimensions and an improvement in left ventricular contractility.

### Anticoagulation management

Prior to the initiation of ECLS, an unfractionated heparin bolus was administered i.v. at a dose of 300 IU/kg. A similar dose was given if the patient had previously been given heparin which had been fully reversed with protamine. If the patient was on cardiopulmonary bypass at the time ECLS was initiated, ECLS was instituted with full heparinisation. Further unfractionated heparin therapy was not administered in the first instance, and protamine sulphate was only administered if surgical bleeding could not be controlled. In the post-operative period, if bleeding was controlled, a continuous intravenous infusion of unfractionated heparin was initiated immediately. A target activated clotting time range of 130–160 seconds was selected, which was measured. For patients with persistent bleeding, for whom a surgical cause had been excluded, heparin was discontinued and not recommenced until the bleeding was under control.

### Statistical analysis

Results of continuous variables are expressed as mean ± standard deviation. For discontinuous variables absolute and relative frequencies are reported. Statistical software SPSS for Windows 21.0 (SPSS Ing, Chicago, IL, USA) was used for data analysis.

## Results

All twelve patients in the study cohort had fulminant cardiogenic shock with lung failure. The underlying cause of refractory cardiogenic shock was acute cardiac decompensation due to dilated cardiomyopathy in three patients (25%), coronary artery disease with acute myocardial infarction (AMI) in three patients (25%) and acute myocarditis in six patients (50%) (Table 2).

**Table 2:** Patient’s characteristics and support strategy

**Patient**	**Diagnosis**	**Age**	**Sex**	**Basic support**	**Support duration (d)**	**Bridged to**
1	DCM	38	male	ECLS with LV vent	4	BiVAD
2	DCM	19	male	ECLS with LV vent	10	BiVAD
3	Myocarditis	15	male	ECLS with LV vent	6	Recovery
4	Myocarditis	12	male	ECLS with LV vent	5	Recovery
5	Acute MI	48	male	ECLS with LV vent	5	BiVAD
6	Acute MI	65	male	ECLS with LV vent	7	BiVAD
7	Acute MI	34	male	ECLS with LV vent	3	BiVAD
8	DCM	37	female	ECLS with LV vent	10	Cardiac transplantation
9	Myocarditis	38	male	ECLS with LV vent	17	Cardiac transplantation
10	Myocarditis	29	male	ECLS with LV vent	17	Cardiac transplantation
11	Myocarditis	20	female	ECLS with LV vent	7	BiVAD
12	Myocarditis	24	male	ECLS with LV vent	7	Recovery

*DCM*, Dilative cardiomyopathy; *MI*, Myocardial infarction; *ECLS*, Extracorporeal life support; *LV*, Left ventricular; *BiVAD*, Biventricular assist device.

All patients required mechanical ventilation with 100% FiO_2_ with a mean peak inspiratory pressure of 32.0 ± 3.57 cmH_2_O and mean positive end-expiratory pressure (PEEP) of 9.9 ± 1.83 cmH_2_O. At the time of ECLS implantation, patients received intravenous adrenaline at a dose of 0.25 ± 0.07 μg/kg/min and noradrenaline at 0.28 ± 0.16 μg/kg/min. On admission, two patients were supported with the CardioHelp™-System (Maquet, Rastatt, Germany), which was upgraded to an ECLS with LV venting. The mean levels of serum creatinine and serum bilirubin before implantation, 24 h after implantation and 3 days after implantation are presented in (Figures 5 and 6). Ten patients had acute liver failure with serum bilirubin levels higher than 20 μmol/L.

**Figure 5:** Perioperative levels of serum bilirubin were significantly lower after 3 days on ECLS support with LV vent (p = 0.001).

**Figure 6:** **Perioperative levels of serum creatinine.** There was a trend towards lower serum creatinine levels after 3 days on ECLS support with LV vent (p = 0.061).

The survival on ECLS support was 100%. All patients were successfully bridged to either recovery (n = 3, 25%), long-term biventricular support (n = 6, 50%) or cardiac transplantation (n = 3, 25%) after mean ECLS support of 8.0 ± 4.3 days (range 3-17 days) (Table 2). The mean cumulative ICU stay (including the stay after ECLS explantation or upgrade) was 23.1 ± 9.6 days. Of all twelve cases, seven patients (58.3%) were discharged from hospital after a mean hospital stay of 42 ± 11.9 days and are currently alive. Three patients recovered on ECLS with no recurrence of cardiac decompensation. The overall survival from ECLS implantation to the end of the study was 58.3%. Four patients died in hospital on ongoing long-term BiVAD support after 60 ± 80.25 days. The cause of death was septic multi-organ-failure in two patients and severe refractory acute respiratory distress syndrome (ARDS) in two patients. One patient died of primary graft failure after successful bridging to transplantation with ECLS, resulting in the need for long-term biventricular assist device (BiVAD) support.

The most frequent postoperative adverse events during ECLS were: coagulation disorder (n = 8, 66.7%); refractory renal failure requiring hemodialysis (n = 6, 50%), surgical re-exploration due to bleeding (n = 5, 41.7%) and cerebrovascular event (ischemic stroke) (n = 1, 8.3%). One deep sternal wound infection at the ECLS side occurred during the postoperative course without affecting outcome.

## Discussion

Inadequate left ventricular decompression and pulmonary edema are recognised limitations of ECLS. Here, we describe a novel technique for decompressing the left ventricle using a modified central ECLS cannulation technique. Blood is drained from the right atrium into the extracorporeal system and is returned to the ascending aorta. To decompress the left ventricle, a large caliber cannula is introduced in the left apex of the left ventricle via the right superior pulmonary vein through the mitral valve and is connected to the ECLS inflow with a Y-connector. This strategy provides decompression of both left and right ventricle in order to give the lungs and the left ventricle a chance to recover by decreasing myocardial oxygen consumption and preserving coronary blood flow. This approach can be used as a “bridge to recovery” and in cases of failed recovery as a “bridge to bridge” until a long-term left ventricular assist device (LVAD) or a biventricular assist device (BiVAD) can be implanted (Figure 7).

**Figure 7:** **Decision-making flowchart: cardiogenic shock and lung failure.** ECMO, extracorporeal membrane oxygenation; LV; left ventricular; LVAD, left ventricular assist device; BIVAD; biventricular assist device.

ECLS provides immediate haemodynamic benefit, both in terms of increased mean and diastolic arterial blood pressure. However, this results in an increased systemic afterload, which in the context of poor left ventricular function may result in impaired left ventricular ejection and persistent aortic valve closure. Severe left ventricular distension can ensue which is potentiated by insufficient right atrial drainage, bronchial and Thebesian venous blood flow, aortic valve insufficiency, and extracardiac left to right shunting. This situation can induce a competitive flow and cause an impaired oxygen supply to the coronary arteries and the cerebral vessels. Elevated left ventricular end-diastolic volume and increased myocardial wall stress results in increased myocardial oxygen demand yet reduced perfusion of the coronary arteries. This mismatch can result in subendocardial ischemia, which can impair myocardial recovery [6,7]. This pathophysiological mechanism can be ameliorated by adequate left ventricular decompression during ECLS.

Furthermore, the absence of direct left ventricular decompression during ECLS under conditions where left ventricular ejection is severely impaired can lead to intraventricular stasis of blood with a resultant risk of thrombus formation. None of our patients showed evidence of left ventricular thrombus during or after ECLS treatment in spite of left ventricular cannulation. Routinely transesophageal echocardiography demonstrated adequate decompression of the left ventricle in all study patients.

In the absence of left ventricular venting, inadequate left ventricular decompression during ECLS can remain undetected for prolonged periods resulting in an elevation of the left-atrial pressure, which can potentially lead to haemoptysis and pulmonary oedema [6]. These complications were not observed in the study cohort. Another advantage of our technique is the ability to perform separate blood gas analyses from both the venous and left ventricular cannula. This allows the monitoring of both recovery of lung function and the timely detection of impaired coronary perfusion under conditions of improved left ventricular function. This problem occurs if, during ECLS the left ventricle starts to eject poorly saturated blood from the lungs into the aortic root resulting in inadequate coronary arterial oxygen saturation. In such circumstances, it is mandatory to increase ventilatory support. It has been shown in an animal model of ECLS with cannulation of the ascending aorta that an adequate oxygen supply of the coronary arteries could only be achieved with high ECLS blood flow rates (85% of calculated maximum) [8]. For that reason, blood gas analysis samples from the left ventricular vent are more informative to those taken from the radial artery.

We believe that continuous monitoring of the cerebral arterial saturation by near-infrared spectroscopy is mandatory for monitoring cerebral perfusion during ECLS. It has been shown that an unregulated increase of the cerebral blood flow increases the risk of spontaneous cerebral haemorrhage during ECLS [9]. Incorrect placement of the aortic cannula in the truncus brachiocephalicus can lead to impaired perfusion of the brain or, at worst, to cerebral oedema and haemorrhage.

Although there are alternative systems for left ventricular unloading like the axial flow Impella® system (Abiomed, Danvers, USA) and the Tandem Heart™ system (CardiacAssist, Pittsburgh, USA), they lack oxygenation capacity and only provide partial unloading of the congested left ventricle. They are deemed unsuitable for patients in refractory cardiogenic shock and respiratory failure [10,11]. Although left ventricular decompression can be achieved via a percutaneous transaortic/transseptal catheter based system, because of the issues described above and the requirement for cannulae of relatively large diameter, central ECLS support with left ventricular decompression is preferred at our institution.

In recent years, portable miniaturized cardiopulmonary bypass/ECMO devices providing up to 10 l/min of blood flow with gas exchange have become available for the treatment of acute cardiogenic shock. The Lifebridge™ (Lifebridge, San Antonio, USA) and CardioHelp™-System (Maquet, Rastatt, Germany) are compact portable ECMO systems. According to the latest AHA-guidelines, these devices are recommended for patients with cardiogenic shock after STEMI who fail to stabilize rapidly with pharmacological therapy alone (class 1/Level of Evidence B) [12]. Two of our study patients were transported to our centre whilst supported with one of these systems (CardioHelp™-System). Support is implemented by puncturing the groin vessels for peripheral veno-arterial ECMO whilst maintaining external cardiac compression. Patients attached to the emergency system can be haemodynamically stabilized thereby allowing diagnostic imaging or can be transferred to specialized centers [13]. A recent meta-analysis of studies using percutaneous circulatory support during high-risk revascularization procedures showed a marked reduction in death of patients in cardiogenic shock (45%) as well as in those who has sustained a cardiac arrest refractory to therapy (40%) [3]. Despite achieving good blood flow rates through these compact systems, some patients do not regain function of either the left ventricle or the edematous lung and this is likely to be attributable, at least in part, to the absence of effective left ventricular decompression.

In the case of peripheral veno-arterial ECMO, if the left ventricle ejects deoxygenated blood into the aorta, there is a risk of cerebral and myocardial hypoxia as a result of the left ventricle selectively perfusing the heart, head and upper limbs whilst the peripheral ECMO perfuses the lower limbs and abdominal organs with oxygenated blood [8]. Myocardial and cerebral hypoxia can go unrecognized [8] and it has been shown that peripheral cannulation is associated with a higher risk of thrombus formation in the aortic root [14].

Peripheral support also necessitates arterial access, with the potential danger of vessel injury and occlusion, which can result in ischemia of the extremities. Cannulation of the neck vessels can lead to injury of the jugular vein or the carotid artery. Foley demonstrated a 21% incidence of extremity ischemia with cannulation of the femoral vessels. These patients were treated with fasciotomy and in one case an amputation had to be conducted [15,16]. Limb ischaemia occurred in none of our patients. The risk of inadequate distal limb perfusion in patients undergoing peripheral cannulation is elevated in those with comorbidities such as peripheral arterial disease and in children [15-17]. Consequently, alternative cannulation sites such as central aortic cannulation and axillary or subclavian artery cannulation should be considered early, to avoid distal limb ischemia.

The fourth annual INTERMACS report [5] revealed that the proportion of INTERMACS level 1 patients has dropped from 42% in 2006, when the database was implemented, to 14% in 2012. Of these patients, only less than 50% of were alive after 12 months [18]. Hence INTERMACS level 1 status (cardiogenic shock) is the greatest risk factor for mortality in VAD therapy [18]. Our study details a patient cohort with severe lung edema and end-organ failure from within and outside the catheter laboratory who were deemed to be candidates for temporary circulatory support. They were not considered suitable for long-term support as weaning from cardiopulmonary bypass would have carried a high risk due to respiratory failure. These patients did not even qualify as INTERMACS level 1 for immediate long-term VAD therapy.

The novel technique described here is believed to confer a significant survival advantage given the dismal prognosis of the study cohort at presentation to our institution. Also important is the timing of device insertion, but this is largely influenced by the timing of referral. Some poor outcomes following ECLS therapy are due to delay in commencing support. Ideally, ECLS should be considered prior to the onset or aggravation of end-organ failure. After initial end-organ recovery with the presented novel technique total artificial hearts with portable consoles may be suitable devices for these patients in future [19,20].

## Conclusion

Our technique highlights the potential use of central ECLS with direct left ventricular decompression in patients with refractory cardiogenic shock and lung failure to facilitate myocardial recovery and prevent pulmonary congestion. Separate blood gas analyses from the venous cannula and the left ventricular vent allow monitoring of pulmonary recovery and facilitate the early detection of coronary hypoxia when the left ventricle begins to recover. Moreover, this strategy is particularly suitable for patients in extremis whose neurologic status is questionable and thus candidacy for cardiac transplantation or long-term support is uncertain. The novel technique described is best suited to centers with established ECLS infrastructure and activity levels, which maintain competency [21-28], [29]. For this reason, regionalization is recommended to ensure that adequate volumes are present at each ECMO center. Given the acuity of care and the risk of sudden decompensation if the circuit fails, intensive specialized staff training is mandatory.

### Consent

Written informed consent was obtained from the patients for publication of this report and any accompanying images.

## Competing interests

The authors declare that they have no competing interests.

## Authors’ contributions

All authors have made substantial contributions to conception and design, or acquisition of data, or analysis and interpretation of data; have been involved in drafting the manuscript or revisiting it critically for important intellectual content and have given final approval of the version to be published. All authors read and approved the final manuscript.
